# The Clinical Efficacy of Cedilanid and Isosorbide Dinitrate plus Pericardial Dissection for Chronic Constrictive Pericarditis in the Elderly and Its Influence on Plasma Endothelin, Atrial Natriuretic Peptide, and Systemic Immune-Inflammation Index

**DOI:** 10.1155/2022/5406649

**Published:** 2022-06-22

**Authors:** Yan Shao, Zhirong Yang, Lu Yin, Qiang Wang, Jie Wang

**Affiliations:** ^1^Department of Cardiovascular Surgery, Qinghai Provincial People's Hospital, Xining, Qinghai, China; ^2^Department of Cardiology, Qinghai Red Cross Hospital, Xining, Qinghai, China; ^3^Department of Hyperbaric Oxygen, Qinghai Provincial People's Hospital, Xining, Qinghai, China; ^4^Department of Anesthesiology, Qinghai Provincial People's Hospital, Xining, Qinghai, China

## Abstract

**Objective:**

To investigate the clinical efficacy of cedilanid and isosorbide dinitrate plus pericardial dissection for chronic constrictive pericarditis in the elderly.

**Methods:**

Ninety elderly patients with chronic constrictive pericarditis admitted to our hospital from March 2018 to October 2020 were recruited and assigned to receive either cedilanid and isosorbide dinitrate (control group A), pericardial dissection (control group B), or cedilanid and isosorbide dinitrate plus pericardial dissection (combination group) via random number table method, with 30 patients in each group. Outcome measures included plasma endothelin, atrial natriuretic peptide, system immune-inflammation indices, treatment effect, quality of life, mental state, and treatment satisfaction.

**Results:**

The combination group had significantly higher treatment satisfaction and treatment efficacy than control groups A and B (*P* > 0.05). The combination group showed the lowest levels of atrial natriuretic peptide and endothelin, followed by control group A, and group B (*P* < 0.001). The combined therapy resulted in significantly lower levels of system immunity index, lower Hospital Anxiety and Depression Scale (HAD) scores, and better General Quality of Life Inventory-74 (GQOLI-74) scores than those of the control group B, followed by group A (*P* < 0.001).

**Conclusion:**

Cedilanid and isosorbide dinitrate plus pericardial dissection for elderly patients with chronic constrictive pericarditis enhances the level of plasma endothelin, atrial natriuretic peptide, and systemic immune-inflammation indexes of patients and improves their quality of life, which shows great potential for clinical promotion.

## 1. Introduction

Chronic constrictive pericarditis is a chronic inflammatory process involving the pericardial wall and visceral layers, causing fibrosis and thickening of the pericardium and limiting the diastolic activity of the heart, thereby reducing cardiac function. The clinical symptoms of chronic constrictive pericarditis are not specific, mainly including progressive dyspnea, fatigue, multiple plasma chamber effusions, edema, cough, weakness, and palpitations [1–3]. Thus, the lack of specific symptoms results in poor early diagnostic outcomes of chronic constrictive pericarditis. With time, myocardial atrophy and fibrosis may occur and lead to a gradual decline of heart function, which significantly compromises the surgical outcomes. At present, pericardial dissection is the treatment of choice for chronic constrictive pericarditis in clinical practice. For some patients with *tuberculosis* in the active stage or intolerance to the operation, conservative treatment with internal medicine is a common practice, but the monotherapy efficiency of either medication or operation leaves much to be desired. The combination of medication and pericardial dissection is marginally explored, and the matching clinical guidance is also insufficient [4–7]. Previous research has shown that the combination of Xuedilan and isosorbide nitrate with traditional Chinese medicine (TCM) decoction is associated with favorable clinical efficacy [8]. In this study, Xuefu Zhuyu decoction was introduced to the patients as adjuvant therapy to treat chronic constrictive pericarditis. The present study analyzed the clinical efficacy of the combination of cedilanid and isosorbide dinitrate plus pericardial dissection for chronic constrictive pericarditis and the effects on plasma endothelin, cardiac natriuretic, and systemic immune-inflammatory indices in patients to provide an experimental basis for subsequent clinical trials.

## 2. Data and Methods

### 2.1. General Data

A total of 90 elderly patients with chronic constrictive pericarditis who were admitted to our hospital from March 2018 to October 2020 were recruited. They were 49 males and 42 females, aged 67.01 ± 3.32 years, with a mean body mass index (BMI) of 27.11 ± 1.59 kg/m^2^, 54 cases of smoking, 63 cases of drinking, 65 cases from urban areas, and 25 cases from rural areas. They were divided into the combination group, the control group A, and control group B via the random number table method with 30 cases in each group. The study design is presented in Figure 1. The sample size was determined using the hospital sample case-control study method with an estimated prevalence of 5% and a relative error of 15% for the sample. With reference to the National Guidelines for the Treatment of Structural Heart Disease risk factor test and other similar large health surveys, the design effect was set at 1.5 with a 95% confidence interval, Za = 1.96, and an incomplete data rate of 10%. The final sample size was set to 30.

### 2.2. Inclusion Criteria

Patients who met the diagnostic criteria for constrictive pericarditis and the diagnosis was confirmed by CT scans or echocardiography, without other organ diseases, infectious diseases, hematological diseases, anesthetic allergies, surgical contraindications, and malignant tumors, and who provided written informed consent were included. This study has been approved by the ethics committee of Qinghai Provincial People's Hospital (approval no. 790771-1).

### 2.3. Exclusion Criteria

Patients who did not meet the inclusion criteria and diagnostic criteria, with valvular heart disease, liver and kidney dysfunction, malignant tumors, blood system disease or infectious disease, severe arrhythmia, allergies to the test drug, and mental illness, were excluded.

## 3. Methods

The patients in control group A received 0.5 mg cedilanid (Shanghai Xudong Haipu Pharmaceutical Co., Ltd.; National Medicine Standard H31021178) diluted in 5% glucose injection daily through intravenous infusion, and isosorbide dinitrate (National Medicine Standard H20065339; Shandong Weifang Pharmaceutical Factory Co., Ltd.) diluted in 5% glucose daily through intravenous infusion.

The control group B received pericardial dissection. With the patient in a supine position general anesthesia was performed, followed by pericardial dissection. A surgical incision was made at the center of the patient's sternum, and the subcutaneous tissue, pectoralis major, and sternum were separated to fully expose the heart, during which important nerves and blood vessels were carefully identified and prevented surgical damage [8, 9]. A resection plan was formulated according to the location and size of the pericardial lesion. After completion of the dissection, electrocoagulation was applied for hemostasis, followed by suturing of the wound. Antibiotics were given to patients after surgery to avoid infection.

The combination group received cedilanid and isosorbide dinitrate plus pericardial dissection, and the treatment regimens were identical to those introduced to the patients in control groups A and B.

### 3.1. TCM Adjuvant Therapy

Chronic constrictive pericarditis mostly involves chest tightness, pain in the anterior region or under the right rib cage, pain with a fixed location or palpitations and shortness of breath, dark tongue or bruised spots, and stringent and astringent pulse. The disease is caused by internal obstruction of blood, so the treatment is to activate blood circulation, resolve stasis, regulate qi, and relieve pain. The Xuefu Zhuyu decoction was introduced as adjuvant therapy for all the patients, and the ingredients include 12 grams of peach kernel, 12 grams of safflower, 15 grams of Chuanxiong Rhizoma, 12 grams of Angelicae Sinensis Radix, 12 grams of red peony, 15 grams of Bupleuri Radix, 10 grams of Aurantii Fructus, 15 grams of Achyranthis Bidentatae Radix, 15 grams of Curcumae Radix, 20 grams of Salviae Miltiorrhizae Radix et Rhizoma, 12 grams of Rhizoma Corydalis, and 12 grams of Platycodonis Radix. Codonopsis Radix and Astragali Radix were added for patients with deficiency of heart qi, Sappan Lignum, Manis Squama, Sparganii Rhizoma, and Curcumae Rhizoma were added for patients with paralysis of the heart, and Asari Radix et Rhizoma and Gui Zhi Ramulus Cinnamomi were added for patients with yin stagnation and severe pain.

### 3.2. Indicators

The “Patient Clinical Satisfaction Questionnaire” prepared by the present department was used to investigate the satisfaction of patients after intervention. The options in the questionnaire are scored on a scale of three levels: fully satisfied, generally satisfied, and dissatisfied. Total satisfaction = fully satisfied rate + generally satisfied rate.

The Generic Quality of Life Inventory-74 (GQOLI-74) [10] was adopted to evaluate the quality of life of the three groups of patients before and after the intervention. The scale includes 4 factors: psychological function, physical function, social function, and material well-being, and the total score is 100 points. The higher the score, the better the quality of life of the patient.

The treatment efficacy of the three groups of patients was statistically analyzed. If the clinical symptoms have been significantly improved, then the treatment is regarded as markedly effective; if the clinical symptoms of the patients have improved, then the treatment effect is regarded as effective; if the clinical symptoms have not been improved or even aggravated, then the treatment is considered ineffective. Total effective rate = markedly effective rate + effective rate.

The Hospital Anxiety and Depression (HAD) scale [11] was used to assess the emotional state of patients before and after the intervention. The scale has a total score of 42 points. The higher the score, the more severe the patient's anxiety and depression.

Radioimmunoassay was used to determine the serum atrial natriuretic factor (ANF) and serum endothelin (ET) levels of the three groups of patients.

The systemic immune-inflammation index (SII) of the three groups of patients was compared. T0 presents patients before the intervention, and T1 and T2 stand for patients at 1 day and 6 days after the intervention, respectively. The systemic immune-inflammation index (SII) of the three groups of patients in different periods was recorded.

### 3.3. Statistical Processing

The data processing software adopted in this study is SPSS20.0, and GraphPad Prism 7 (GraphPad Software, San Diego, USA) was used to plot the graph. The count data are expressed as rates (%) and analyzed using the chi-square test. The measurement data are expressed as (mean ± standard deviation) and analyzed using the chi-square test. One-way ANOVA was used for intergroup comparison. Statistically significant results were defined as *P* < 0.05.

## 4. Results

### 4.1. Baseline Characteristics

There were no significant differences in the baseline characteristics such as age, gender, BMI, smoking, drinking, and place of residence between the three groups of patients (*P* < 0.05), as listed in Table 1.

### 4.2. Treatment Satisfaction

The combination group showed significantly a higher satisfaction rate than control group B, followed by control group A (*P* < 0.05), as listed in Table 2.

### 4.3. Treatment Efficacy

The combined therapy used in the combination group resulted in significantly higher treatment efficacy than the control group B, followed by control group A (*P* < 0.05), as listed in Table 3.

### 4.4. ANF Levels

The combination therapy was associated with more reduction in the levels of ANF versus the monotherapy of either medication or surgery (*P* < 0.001), as shown in Figure 2.

### 4.5. ET Levels

The combination group had a lower level of ET, followed by control group B and then group A (*P* < 0.001), as shown in Figure 3.

### 4.6. GQOLI-74 Scores

The combination group showed the highest GQOLI-74 scores, followed by the control group B and then control group A (*P* < 0.001), as shown in Figure 4.

### 4.7. HAD Scores

The combination group had the lowest HAD scores, followed by the control group B and then control group A (*P* < 0.001), as shown in Figure 5.

### 4.8. SII Scores

There was no significant difference in SII between the three groups of patients before the intervention (*P* > 0.05). The SII of the combination group was significantly lower than that of the control group B, followed by the control group A at 1 and 6 days after the intervention (*P* < 0.001), as shown in Figure 6.

## 5. Discussion

The pericardium has a protective effect on the heart, preventing excessive enlargement of the heart chambers to maintain a constant blood volume. The cardiac output of patients with chronic constrictive pericarditis decreases, and the stroke volume is also reduced. In patients with more severe constrictive pericarditis or those who are physically active, the heart rate will increase to maintain cardiac output, which may predispose them to other serious diseases [12–16]. Related studies have shown that the main cause of chronic constrictive pericarditis is idiopathic or viral pericarditis. In addition, radiation therapy and surgery, *tuberculosis*, and the application of immunosuppressive agents may be major contributors to the development of the disease. Currently, the treatment of constrictive pericarditis remains a key clinical concern [17–21]. Surgery is the mainstay of treatment for constrictive pericarditis, but its efficacy remains mediocre. The present study used cedilanid and isosorbide dinitrate plus pericardial dissection to treat patients with chronic constrictive pericarditis and achieved significant therapeutic effects.

Studies have found that atrial natriuretic peptide is a hormone secreted by the atria and plays a role in natriuretic regulation, diuresis, vasodilation, and blood pressure reduction. Atrial natriuretic peptide involves in the body's water and salt metabolism and regulates cardiovascular function [22–24]. Endothelin, as an active peptide with biological activity, has been reported in relevant studies to be the most potent vasoconstrictor peptide to date. The results of the present study showed that the atrial natriuretic peptide level and endothelin level of the combination were significantly lower than those of the control groups (*P* < 0.05). It is consistent with the research results of Goldstein and Kern [25]. The results showed that after the intervention, the atrial natriuretic peptide levels in the combination group, control group B, and control group A were (236.79 ± 41.27) ng/L, (251.76 ± 59.62) ng/L, and (299.15 ± 88.37) ng/L, respectively; the endothelin in the combination group, control group B, and control group A were (29.77 ± 10.61) ng/L, (38.04 ± 11.13) ng/L, and (47.96 ± 14.66) ng/L (*P* < 0.05), respectively. Presumably, the reasons might be as follows: (1) after pericardial dissection, the enhanced cardiac function decreases the level of ANF, and the level of ET positively correlates with the impairment of cardiac function and interacts with ANF to regulate vasoconstriction and diastole; (2) cedilanid inhibits Na + -K+ active coupling transport inside and outside the cardiomyocyte membrane, increases Na + content in cardiomyocytes, improves myocardial contractility and cardiac hemodynamic status, elevates cardiac output, eliminates the reflex increase in sympathetic tone, thereby mitigating the serum ANF and ET levels. (3) Isosorbide dinitrate releases nitric oxide to relieve vascular smooth muscle dilation and cardiac stress and reduce myocardial oxygen consumption, thereby enhancing cardiac function and affecting serum ANF and ET levels. The results of the present study showed that all three methods were effective in the treatment of elderly patients with chronic constrictive pericarditis, and their combined use potentiates the treatment efficiency. Traditional Chinese medicine is characterized by its holistic concept related to the five viscera and treats chronic constrictive pericarditis in terms of blood stasis, thus achieving blood activation and stasis dissolution. The combination of TCM with western medicine and surgery contributes to faster postoperative recovery in elderly patients with chronic constrictive pericarditis.

## 6. Conclusion

The efficacy of the present study is definite, and the data are reliable. Cedilanid and isosorbide dinitrate plus pericardial dissection for elderly patients with chronic constrictive pericarditis. It effectively improves the levels of plasma endothelin, atrial natriuretic peptide, and systemic immune-inflammation indices, eliminates the patient's negative emotions, and enhances their satisfaction with treatment. The limitations of this single-centered article are the lack of long-term follow-up data and the small sample size. Future multicenter studies will be conducted to extend the study length and expand the included sample size to obtain more reliable clinical data.

## Figures and Tables

**Figure 1:** Study design.

**Figure 2:** Comparison of ANF scores among the three groups ( ¯*x* ± *s*) Note: the abscissa indicates before and after the intervention, and the ordinate indicates the ANF score, ng/L. The ANF levels of patients in control group A before and after intervention were (419.68 ± 110.13) ng/L and (299.15 ± 88.37) ng/L, respectively. The ANF levels before and after intervention in control group B patients were (418.57 ± 109.42) ng/L and (251.76 ± 59.62) ng/L, respectively. The ANF levels of (419.35 ± 110.05) ng/L and (236.79 ± 41.27) ng/L before and after the intervention in the combination group patients, respectively. A significant difference in ANF levels in the control A group compared to the control B group after the intervention (*t* = 8.980, ^*∗∗∗*^*P* < 0.001). Asignificant difference in ANF levels in the control B group compared to the combination group post-intervention (*t* = 5.726, ^*∗∗∗*^*P* < 0.001). A significant difference in ANF levels in the control A group compared with the combination group after the intervention (*t* = 2.982, ^*∗∗∗*^*P* < 0.001).

**Figure 3:** Comparison of ET scores among the three groups ( ¯*x* ± *s*) Note: the abscissa denotes before and after intervention, and the ordinate denotes ET score, ng/L. The ET levels of patients in control group A before and after intervention were (67.14 ± 21.68) ng/L and (47.96 ± 14.66) ng/L, respectively. The ET levels of patients in the control group B before and after the intervention were (66.73 ± 21.46) ng/L and (38.04 ± 11.13) ng/L, respectively. The ET levels of patients in the combined group before and after intervention were (66.95 ± 21.53) ng/L and (29.77 ± 10.61) ng/L, respectively. A significant difference in the comparison of ET levels between control group A and control group B after intervention (*t* = 7.961, ^*∗∗∗*^*P* < 0.001). A significant difference between the control B group compared with the combination group in terms of post-intervention ET levels (*t* = 4.916, ^*∗∗∗*^*P* < 0.001). A significant difference in the comparison of ET levels after intervention between the control A group and the combination group (*t* = 3.615, ^*∗∗∗*^*P* < 0.001).

**Figure 4:** Comparison of GQOLI-74 scores among the three groups ( ¯*x* ± *s*) Note: The abscissa denotes before and after the intervention and the ordinate denotes GQOLI-74 score, points. The GQOLI-74 scores before and after intervention for patients in control group A were (46.72 ± 7.43) and (61.25 ± 4.22), respectively. The GQOLI-74 scores of patients in control group B before and after intervention were (46.44 ± 7.88) and (78.33 ± 4.98), respectively. The GQOLI-74 scores of patients in the combined group before and after intervention were (46.53 ± 7.61) and (90.35 ± 5.67), respectively. A significant difference in GQOLI-74 scores compared between the control A group and the control B group after the intervention (t = *t* = 25.828, ^*∗∗∗*^*P* < 0.001). A significant difference in GQOLI-74 scores compared between the control B group and the combined group after the intervention (*t* = 11.407, ^*∗∗∗*^*P* < 0.001). A significant difference in GQOLI-74 scores comparing the control A group with the combination group after the intervention (*t* = 21.663, ^*∗∗∗*^*P* < 0.001).

**Figure 5:** Comparison of HAD scores among the three groups ( ¯*x* ± *s*) Note: the abscissa denotes before and after the intervention, and the ordinate denotes the HAD score, in points. The HAD scores of patients in control group A before and after intervention were (35.88 ± 3.22) and (13.29 ± 2.53), respectively. The HAD scores of patients in control group B before and after intervention were (35.81 ± 3.25) and (7.56 ± 1.49) points, respectively. The HAD scores of patients in the combination group before and after the intervention were (35.79 ± 3.34) and (4.67 ± 1.01), respectively. A significant difference in HAD scores between control group A and control group B after the intervention (*t* = 58.901, ^*∗∗∗*^*P* < 0.001). A significant difference in HAD scores between the control B group and the combination group after the intervention (*t* = 37.005, ^*∗∗∗*^*P* < 0.001); A significant difference in HAD scores between the control A group and the combination group after the intervention (*t* = 18.968, ^*∗∗∗*^*P* < 0.001).

**Figure 6:** Comparison of HAD scores among the three groups ( ¯*x* ± *s*) Note: the abscissa denotes the T0, T1, and T2 time points, respectively, and the ordinate denotes SII. The SII at T0, T1, and T2 for patients in control group A were (495.14 ± 20.19), (501.64 ± 20.57), and (486.34 ± 20.47), respectively. The SII at T0, T1 and T2 for patients in control group B were (495.13 ± 20.18), (442.09 ± 20.61) and (413.47 ± 20.51), respectively The SII at T0, T1 and T2 for patients in the combined group were (495.07 ± 19.86), (399.72 ± 18.65) and (363.51 ± 17.77), respectively. A significant difference in SII at T1 among the three groups of patients (*t* = 13.719, ^*∗∗∗*^*P* < 0.001). A significant difference in SII at T2 among the three groups of patients (*t* = 16.869, ^*∗∗∗*^*P* < 0.001).

**Table 1:** Comparison of general data of the three groups of patients [n (%)].

	Control group B (*n* = 30)	Control group A (*n* = 30)	Combination group (*n* = 30)	x^2^ or t	*P*
Age (year)				0.086	0.932
	66.75 ± 3.32	66.69 ± 3.29	65.97 ± 3.24		

Gender				0.178	0.673
Male	16	15	17		
Female	14	15	13		

BMI (kg/m2)				1.119	0.266
	26.27 ± 1.59	25.89 ± 1.63	25.91 ± 1.58		

Smoking				0.030	0.832
Yes	18	17	19		
No	12	13	11		

Drinking				0.178	0.673
Yes	20	21	22		
No	10	9	8		

Place of residence				0.050	0.822
Urban	21	22	22		
Rural	9	8	8		

**Table 2:** Comparison of satisfaction among the three groups.

Groups	n	Highly satisfied	Satisfied	Dissatisfied	Total satisfaction(%)
Control group A	30	13	9	8	22 (73.33)
Control group B	30	18	8	4	26 (86.67)
Combination group	30	22	7	1	29 (96.67)
x^2^					6.480
*P*					0.011

**Table 3:** Comparison of treatment efficacy among the three groups.

Groups	n	Markedly effective	Effective	Ineffective	Total effectiveness (%)
Control group A	30	13	11	6	22 (80.33)
Control group B	30	18	9	3	26 (90.00)
Combination group	30	23	6	1	29 (96.67)
x^2^					6.049
*P*					0.014

## Data Availability

The datasets used during the present study are available from the corresponding author upon reasonable request.
